# Effect of the Influenza Virus Rapid Antigen Test on a Physician's Decision to Prescribe Antibiotics and on Patient Length of Stay in the Emergency Department

**DOI:** 10.1371/journal.pone.0110978

**Published:** 2014-11-06

**Authors:** Hye Won Jeong, Jung Yeon Heo, Jung Soo Park, Woo Joo Kim

**Affiliations:** 1 Department of Internal Medicine, Chungbuk National University College of Medicine, Heungduk-gu, Cheongju, Republic of Korea; 2 Department of Emergency Medicine, Chungbuk National University College of Medicine, Heungduk-gu, Cheongju, Republic of Korea; 3 Division of Infections Disease, Department of Internal Medicine, Korea University College of Medicine, Guro-dong, Guro-gu, Seoul, Republic of Korea; 4 Transgovernmental Enterprise for Pandemic Influenza in Korea, Seoul, Republic of Korea; University of Hong Kong, Hong Kong

## Abstract

**Background:**

Influenza virus infection is a common reason for visits to the emergency department (ED) during the influenza season. A rapid and accurate diagnosis of influenza virus infection is important to reduce unnecessary antibiotic prescription and to improve patient care. The aim of this study was to examine whether using the Influenza Virus Rapid Antigen Test (IVRAT) in the ED affects the decision to prescribe antibiotics or the length of hospital stay (LOS).

**Methods:**

Data from patients suffering from an influenza-like illness (ILI) and who were discharged after visiting the ED at Chungbuk National University Hospital were reviewed over two influenza seasons: 2010–2011, when IVRAT was not used in the ED, and 2011–2012, when it was. The numbers of antibiotic prescriptions issued and the ED LOS during these two seasons were then compared.

**Results:**

The number of antibiotic prescriptions was significantly lower in 2011–2012 (54/216, 25.0%) than in 2010–2011 (97/221, 43.9%; *P*<0.01). However, the median ED LOS for patients in 2011–2012 was much longer than that of patients in 2010–2011 (213 minutes *vs*. 257 minutes; *P*<0.01). During the 2011–2012 influenza season, 73 ILI patients showed a positive IVRAT result whereas 123 showed a negative result. Upon discharge, antibiotics were given to 42/123 (34.1%) ILI patients with a negative IVRAT result, but to only 7/73 (9.6%) patients with a positive IVRAT result (*P*<0.01).

**Conclusions:**

Performing IVRAT in the ED reduced the prescription of antibiotics to ILI patients discharged after ED care. However, the ED LOS for patients who underwent IVRAT was longer than that for patients who did not. Thus, performing IVRAT in the ED reduces the unnecessary prescription of antibiotics to ILI patients during the influenza season.

## Introduction

Influenza virus infection is a common reason for visits to the emergency department (ED) during annual influenza epidemics. The incidence of medically-attended illness (influenza-like illness (ILI) severe enough to cause the patient to seek medical care) in unvaccinated populations is estimated to be 10–20%, although the rates can be as high as 40–50% [1]–[3]. Non-specific symptoms such as high fever and a rapid deterioration in the patients' general condition mean that the clinical manifestations of influenza virus infection may mimic bacterial sepsis, particularly in young infants and the elderly [4], [5]. A diagnosis of influenza can be made by viral culture or by RT-PCR analysis of nasal or throat swab specimens [6], [7]. Various techniques are also available for the rapid diagnosis of influenza at the point-of-patient care [8]. Most are based on specific antibodies that detect viral antigens in respiratory secretions. The test results are visualized on a filter paper, an optical device, or a dipstick.

The rapid and specific diagnosis of influenza virus infection in the ED is important for optimal patient care and infection control, since patients can then receive appropriate antiviral therapy. The influenza virus rapid antigen test (IVRAT) is valuable in the ED setting because it is simple to perform and has a fast turnaround time. However, it has low sensitivity (40–80%) though its specificity is very high [9], [10]. Despite this, some small studies of pediatric ILI patients show that a positive IVRAT test results in a fall in the number of antibiotic prescriptions issued in the ED, reduces the need for additional diagnostic tests, and reduces the ED length of stay (LOS) [11]–[13]. However, a large systematic review of pediatric patients in the ED showed that the routine use of IVRAT had no significant effect on the rate of antibiotic prescription; it also showed that even though patients that received IVRAT were less likely to undergo chest radiography, the ED LOS was no different [14].

It is not clear whether the use of IVRAT in the ED affects a physician's decision making. No studies have examined whether testing adult ILI patients with IVRAT reduces antibiotic prescription and ED LOS. Therefore, the aim of this study was to examine the effect of IVRAT on the prescription of antibiotics and ED LOS in adult ILI patients.

## Materials and Methods

### Study design and patient population

Chungbuk national university hospital, a 620-bed teaching hospital in Cheongju, Republic of Korea, began performing IVRAT in the ED during the 2011–2012 influenza season, when it became a participant in a sentinel hospital-based surveillance system for influenza (Hospital-based Influenza Morbidity and Mortality; HIMM) [15]. During the 2011–2012 season, all ILI patients who visited the ED were encouraged to provide consent for IVRAT. Nasal or throat swab specimens from ILI patients managed in the ED were tested at the bedside using influenza detections kits (SD Bioline Influenza Antigen Test, Standard Diagnostics, Kyonggi, Korea). At the same time, an additional swab specimen was taken and transported to the central HIMM laboratory. ILI was defined as the presence of fever (temperature ≥38°C, as measured in the ED) accompanied by at least one of the following respiratory symptoms (recorded by the attending physician): cough, sore throat, or rhinorrhea [15].

The medical records of ILI patients who visited the ED at Chungbuk National University Hospital during the 2010–2011 (pre-IVRAT) and 2011–2012 (IVRAT) influenza seasons were reviewed by infectious disease specialists. The following data were collected: the patients' reason for visiting the ED; the medical diagnosis made by the ED primary physicians; the time of arrival at the ED; the time at which the patient was seen by an ED physician; the decision regarding whether to hospitalize the patient; and the time at which the patient was discharged from the ED. If the patient was discharged home after ED care, the patient's discharge medications were also reviewed. The influenza season was roughly defined as the period from November to February. All ILI patients discharged from hospital after ED care were included in the study. The rates of antibiotic prescription and ED LOS (the time interval between the patient being seen by the physician and their departure from the ED) during each of the two influenza seasons were then compared. The characteristics of ILI patients with a positive IVRAT result and of those with a negative result were also compared.

Patients hospitalized after ED care were excluded from the study. This is because the most common reason for hospitalization was pneumonia, which requires treatment with antibiotics (in most cases). Another reason is because other factors, such as waiting for an available room on the ward, would affect the ED LOS for this group.

### Ethics statement

The study protocol was approved by the Institutional Review Board of Chungbuk National University Hospital (IRB No. 2012-02-012) and all participants (or next of kin/caregiver in the case of children) who attended the ED during the 2011–2012 (IVRAT) season provided written informed consent to their participation in the study. Consent was waived in the case of ILI patients attending the ED during the 2010–2011 (pre-IVRAT) season. Patient records were anonymized and de-identified prior to analysis.

### Statistical analysis

Categorical variables were compared using the Chi-squared or Fisher's exact tests. Continuous variables that did not show a normal distribution were compared using the Mann-Whitney test. SPSS version 13.0 (SPSS, Inc., Chicago, IL) was used for all statistical analyses. All tests were two-tailed. A *P* value <0.05 was considered statistically significant.

## Results

During the 2010–2011 influenza season, 493 ILI patients visited the ED at Chungbuk National University Hospital. Of these, 221 were discharged after ED care (group A) and 264 were hospitalized. During the 2011–2012 influenza season (when the hospital began using IVRAT in the ED), 448 ILI patients visited the ED and 216 patients were discharged after ED care (group B). Data from the patients who were discharged after ED care in each year (groups A and B) were analyzed and the results were compared (Figure 1).

**Figure 1:** ILI patients examined in the present study. A. 2010–2011 influenza season (pre-IVRAT year). B. 2011–2012 influenza season (IVRAT year).

The age-range of the patients in group A was from newborn to 88 years and that of group B was from newborn to 100 years. The median age of the patients group B was greater than that of patients in group A (9.0 years *vs.* 34.5 years, respectively; *P*<0.01), and 47.5% (105/221) of the patients in group A and 54% (117/216) in group B were female. Antibiotics were prescribed to 97 patients (43.9%) in group A and to 54 patients (25.0%) in group B (Table 1). Thus, the proportion of antibiotic prescription was significantly lower in 2011–2012 than in 2010–2011 (*P*<0.01). ILI patients were most often prescribed cephalosporins and amoxicillin/clavulanate (Table 2). The median ED LOS for patients in group B was much longer than that of patients in group A (213 minutes *vs*. 257 minutes; *P*<0.01; Table 1). The overall ED LOS of all patients who visited ED was not significantly different between the two seasons (median 152 minutes vs. 156 minutes; *P* = 0.35).

**Table 1:** The average length of stay and antibiotic prescription rates for patients with influenza-like illness discharged after emergency department care during the 2010–2011 and 2011–2012 influenza seasons.

	Group A (n = 221)	Group B (n = 216)			*P* value
		IVRAT-positive (n = 73)	IVRAT- negative (n = 123)	IVRAT not performed (n = 20)	
Proportions of antibiotic-prescribed patients (%)	97/221 (43.9)	54/216 (25.0)			*P*<0.01
		7/73 (9.6)	42/123 (34.1)	5/20 (25.0)	*P*<0.01
Median ED LOS (min) (range)	213 (11–1464)	257 (16–1755)			*P*<0.01

Abbreviations: ED, emergency department; IVRAT, influenza virus rapid antigen test; LOS, length of stay; n, number.

**Table 2:** Antibiotics prescribed to patients discharged after ED care during the two influenza seasons.

Antibiotic	2010–2011 influenza season	2011–2012 influenza season
Cephalosporins	53	21
Amoxicillin/clavulanate	38	18
Quinolones	3	13
Macrolides	3	2
Total	97	54

Next, we examined the number of antibiotic prescriptions and ED LOS in group B patients according to the IVRAT results. Of the 216 patients eligible for testing, 73 showed a positive result and seven (9.6%) were prescribed antibiotics; however, antibiotics were prescribed to 42/123 (34.1%) of the ILI patients with a negative IVRAT result. Of the 20 patients who refused the IVRAT test, five received antibiotics (25.0%). Thus, a positive IVRAT result led to a significant reduction in the number of antibiotics prescriptions issued (*P*<0.01; Table 1). The median ED LOS for the 73 patients with a positive IVRAT result was 265 minutes, which was longer than (but not significantly different from) that of the 123 patients with a negative IVRAT result (253 minutes; *P* = 0.15).

## Discussion

Here, we examined whether performing IVRAT in the ED affected the number of antibiotic prescriptions issued to ILI patients discharged home after ED treatment. We also examined whether IVRAT had an effect on the ED LOS for these patients. We found that performing IVRAT in the ED reduced the number of antibiotics prescriptions issued to ILI patients who were not hospitalized. However, the ED LOS for ILI patients discharged home after ED care was actually longer during the influenza season in which IVRAT was performed than in the previous season when IVRAT was not performed. Taken together, these findings suggest that IVRAT affects a physician's decision making and reduces the prescription of antibiotics to ILI patients.

A diagnosis of influenza can be made on epidemiologic grounds. When the influenza virus is known to be circulating within a community, predictive clinical symptoms and signs are diagnostic in around 80% of cases [16]–[18]. The most reliable predictive symptoms are acute fever and cough [17]. Due to the high accuracy of a clinical diagnosis and the relatively low sensitivity of IVRAT, some believe that IVRAT is not necessary in clinical settings that utilize local influenza surveillance systems. However, the present study clearly shows that performing IVRAT in the ED led to a reduction in the number of antibiotics prescriptions issued to non-hospitalized ILI patients by ED physicians. This suggests that IVRAT can play an important role in distinguishing true influenza patients from those with other acute febrile illnesses. Making a clinical diagnosis of influenza during the annual influenza season is not difficult for specialists in infectious or respiratory disease, even in the absence of laboratory tests. However, it can be difficult in the ED setting, which is usually overcrowded and in which ILI patients without complications are usually triaged and are regarded as “less-urgent” than other patients [19]. The present study shows that performing IVRAT in the ED can improve influenza diagnosis and reduce the unnecessary prescription of antibiotics. Although we did not review patient data regarding the prescription of antiviral medicines, a previous study shows that a positive IVRAT test results in the early treatment of influenza patients with appropriate antiviral medicines [11].

Some studies show that prescribing antibiotics to patients with upper respiratory infections prevents secondary infectious complications and reduces the severity of symptoms [20], [21]. However, considering the possible adverse effect of antibiotics and their role in the development of antibiotic resistance, the benefit derived from prescribing antibiotics for upper respiratory infections is probably very small. Indeed, a previous study shows that immediate prescription of antibiotics to treat uncomplicated upper respiratory infections is not associated with better clinical outcomes or improved patient satisfaction when compared with delayed or no treatment [22]. However, we found that antibiotics were prescribed to 43.9% of ILI patients in group A and to 25.0% of ILI patients in group B. This high percentage of antibiotics prescription may be related to patients' expectations and/or to concerns about secondary infectious complications. We believe that further study of antibiotics prescription in the ED is necessary to reduce usage in this setting.

LOS is an important variable to consider when evaluating the quality and efficacy of ED care. Most hospitals make a huge effort to reduce ED LOS. The results of the present study show that the ED LOS was actually longer when IVRAT was performed in the ED. The reasons of this are not clear. ED LOS is influenced by many factors, including a shortage of hospital beds, overcrowding, patient admission and discharge procedures, and the speed at which the ED physicians work [23], [24]. Thus, it may be that factors other than IVRAT led to the increase in ED LOS observed for group B. Another consideration is that the mean age of the patients in group B was higher than that in group A; therefore, these patients may have had comorbidities that increased the work-up time in the ED. The overall ED LOS of all patients who had visited ED was not significantly different between the two seasons. Although the actual time taken to get informed consents and perform IVRAT to ILI patients was not so long, that may be one reason of longer ED LOS in 2011–2012 season. Further studies are needed to clarify this.

The present study is the first to examine the effects of IVRAT on antibiotic prescription and ED LOS in adult ILI patients. In contrast to a large meta-analysis of pediatric ILI patients, which showed that IVRAT had no effect on antibiotic prescription to ILI patients [14], we found that IVRAT reduced the number of antibiotic prescriptions issued to influenza patients who were discharged home from the ED. The design of the present study is different from that of other studies that compared data from IVRAT-positive and IVRAT-negative patients [13], or compared data from patients in whom IVRAT was performed with those from patients in whom IVRAT was not performed during the same influenza season [11]. The design of these studies may introduce bias by only performing IVRAT on patients who showed clear clinical symptoms and signs of influenza; therefore, the results might not represent the true effects of IVRAT on a physician's decision making. The results of the present study provide a more accurate picture of how IVRAT affects the decision to prescribe antibiotics.

In summary, performing IVRAT in the ED reduces the number of antibiotic prescriptions issued to ILI patients discharged home after ED care. Also, IVRAT is very useful for differentiating influenza from other acute febrile illnesses. These findings suggest that widespread use of IVRAT in the ED will reduce the unnecessary prescription of antibiotics to ILI patients during influenza seasons, which is important in a climate of increasing antibiotic resistance.
